The article "Clinical Observation of Fuzheng Xiaoji Granule in the Treatment of Stage IIIC Colorectal Cancer" was published in 2022. Journal: Evid Based Complement Alternat Med.

# Clinical Observation of Fuzheng Xiaoji Granule in the Treatment of Stage IIIC Colorectal Cancer

**DOI:** 10.1155/2022/4618342

**Published:** 2022-09-21

**Authors:** Lingling Lv, Xiaoheng Shen, Jun Zhang, Qiong Li, Junwei Wu, Yuan Wu, Jingxian Chen, Wenhua Zhu, Lan Zheng

**Affiliations:** ^1^Department of Traditional Chinese Medicine, Ruijin Hospital, Shanghai Jiaotong University School of Medicine, Shanghai 200025, China; ^2^Department of Oncology, Ruijin Hospital, Shanghai Jiaotong University School of Medicine, Shanghai 200025, China

## Abstract

**Objective:**

This study aimed to evaluate the effectiveness and safety of Fuzheng Xiaoji granule in patients with stage IIIC colorectal cancer.

**Methods:**

A total of 150 patients with stage IIIC colorectal cancer treated in Shanghai Ruijin Hospital from January 2019 to January 2022 were selected. They were divided into treatment and control groups according to a 2 : 1 random number table. There were 100 cases in the treatment group and 50 cases in the control group. The treatment group was administered Fuzheng Xiaoji (FZXJ) granule, and the control group was administered the placebo orally. The primary endpoint was disease-free survival (DFS). In addition, after 6 months, the changes in Traditional Chinese Medicine (TCM) symptom score (fatigue, emotional depression, chest tightness, insomnia, anorexia, abdominal distension, abdominal pain, soreness and weakness in the waist and legs, chills, and dysphoria in the chest, palm, and soles) were compared.

**Results:**

The DFS was 34.37 ± 2.91 months in the control group and 37.0 ± 1.08 months in the treatment group (*p* < 0.05). Compared with the control group, the treatment group showed less fatigue, abdominal distension, and soreness and weakness in the waist and legs (*p* < 0.05), significantly. The scores of emotional depression and anorexia decreased obviously, with a significant difference between the control and treatment groups (*p* < 0.01). There were no significant differences between the control and treatment groups in the incidence of chest tightness, insomnia, abdominal pain, chills, and dysphoria in the chest, palm, and soles (*p* > 0.05).

**Conclusion:**

Fuzheng Xiaoji granule can improve patients' symptoms and prolong the DFS.

## 1. Introduction

### 1.1. Colorectal Cancer

Colorectal cancer is the third most common cancer in the world. According to the cancer data statistical report published by CA magazine in 2021, about 160,000 people in the United States were newly diagnosed with colorectal cancer [1], while the situation of colorectal cancer in China is complicated. The latest prediction is that, in China, there will be about 592,200 new cases in 2022, accounting for 12.6% of all cancer cases [2]. Nearly 60% of patients are in the late stage of disease at the time of diagnosis and have already missed the opportunity for a radical cure. The 5-year survival time of patients with stage IIIC colorectal cancer is only 27%-44% [3, 4]. Due to a large number of patients with colorectal cancer, the number of stage IIIC patients should not be underestimated. Additionally, stage IIIC colorectal cancer has a poor prognosis. Therefore, it is necessary to find a method to reduce the toxicity and increase the efficiency of chemotherapy drugs to promote body recovery and improve overall prognosis. Surgery is the primary method used to treat colorectal cancer, but the 5-year survival rate of patients with colorectal cancer treated by surgery alone is only about 50%. About 40%-50% of patients experience recurrence or metastasis after the operation, and most patients lose the chance of being recured [5]. Therefore, finding effective postoperative adjuvant therapy to inhibit tumor metastasis, thereby improving the DFS and prolonging the survival time, has long been the focus of oncologists.

Stage III colorectal cancer is the primary and absolute indication for adjuvant chemotherapy and is also the primary beneficiary of adjuvant chemotherapy. Therefore, improving the DFS rate of these patients is of great clinical significance. At present, modern medicine has no suitable treatment. Therefore, it is indispensable to use TCM to improve the side effects of chemotherapy and significantly prolong the DFS. Since the guidelines still have no effective means to prolong the DFS of colorectal cancer patients after adjuvant chemotherapy, further reducing the risk of recurrence based on postoperative adjuvant chemotherapy has become one of the essential tasks of the medical community. In this study, we focus on TCM's synergistic, auxiliary, and regulatory effects on these patients. We also explore the postadjuvant chemotherapy treatment mode of integrated traditional Chinese and Western medicine. It is imperative to devise an integrated traditional Chinese and modern medicine treatment strategy, in which TCM reduces the toxicity of chemotherapy drugs and increases their effectiveness against tumor cells.

### 1.2. Traditional Chinese Medicine

TCM has a long history. Since ancient times, treating malignant tumors based on syndrome differentiation has effectively improved the quality of life and prolonged survival, which has been widely appreciated in China and abroad. Many studies on colorectal cancer [6–8] have shown that TCM has unique advantages in reducing the toxic and side effects of chemotherapy, improving quality of life, and regulating body immunity.

According to the incidence and clinical characteristics of colorectal cancer, ancient books of TCM attribute it to “intestinal wind,” “anal hemorrhoids,” “internal hemorrhoids,” “lumps and bumps,” and other disease syndrome categories. According to TCM theory, a deficiency of vital-*qi* is not just the internal basis for the occurrence of various tumors, it is also the root cause; as the ancient Chinese text “*Su Wen*” says, “when there issufficient vital-*qi inside*, and evil cannot invade the health body.” (“*Zheng qi cun nei, xie bu ke gan*“). This means that if an individual has a strong immune system, then elements of the external environment, such as bacteria and viruses, will not make them sick. Another ancient Chinese text, “Synopsis of the Golden Chamber,” says that “Zang-Fu organs, meridians, and collaterals have successively suffered from disease and pulse syndrome” and “if the five internal organs are smooth, people will be healthy.” This means that as long as the organs function properly, the body will be healthy. According to the compilation of surgical medical records, “deficiency in healthy-*qi* leads to bumps (“Yan” in TCM, the same as cancer).” Therefore, the deficiency of vital energy and the imbalance of *yin* and *yang* in the internal organs and viscera (Zang-Fu organs) are the leading internal causes of tumors. Therefore, in line with this pathogenesis, Professor Xiaoheng Shen, a well-known TCM doctor in Shanghai, developed a method for strengthening and eliminating the accumulation of bumps and lumps—the Fuzheng Xiaoji theory [9–12].

Professor Xiaoheng Shen formulated the method of strengthening the vital energy and eliminating accumulation combined with the differentiation of disease and syndrome. She also formulated her prescription by stages (the radiotherapy and chemotherapy stage, rehabilitation stage, and tumor progression stage). Furthermore, in addition to containing the main drug, the prescription includes some auxiliary drugs to treat the accompanying symptoms. This study used the basic prescription of the FZXJ method in the rehabilitation period for clinical observation.

## 2. Materials and Methods

### 2.1. Study Design

This study was a prospective, randomized, nondouble-blind, single-center, clinical study. The study design is shown in Figure 1. A total of 150 patients with colorectal cancer, under the guidance of FZXJ therapy and using the random number table method, were divided into the TCM FZXJ treatment group and the placebo control group in a 2 : 1 ratio; that is, 100 cases were in the treatment group and 50 cases were in the control group. The DFS between the two groups was compared, and the change in TCM syndrome score was evaluated.

### 2.2. Ethical Approval

The Ethics Committee of Ruijin Hospital, Affiliated with Shanghai Jiao Tong University School of Medicine, approved the study on December 29, 2018. The approval number was the 2018 provisional ethical review (No. 222). The project was registered at the China Clinical Trial Registry on April 24, 2019 (registration number, ChiCTR1900022755; registration title: Application Value of Fuzhong Xiaoji Therapy after Adjuvant Treatment of Stage IIIC Colorectal Cancer). The final official trials began on May 5, 2019, and ended on February 28, 2022. This study followed the principles of the Helsinki Declaration and the guidelines for good clinical practice. Informed consent was obtained from the enrolled patients.

### 2.3. Determination of the Sample Size

With a test efficiency of 80%, an alpha of 0.2, an HR of 0.4135, and an abscission rate of 10%, the required sample size would be 148; with an abscission rate of 5%, the sample size would be 140, and with an abscission rate of 0%, the sample size would be 133. Therefore, the total number of samples required was 133-148. According to the new measured value, the sample size was expanded from 120 to 150, including 50 cases in the control group and 100 cases in the treatment group.

### 2.4. Study Population

One hundred and fifty patients with stage IIIC colorectal cancer were randomly divided into the TCM treatment group and the placebo control group in a 2 : 1 ratio after completing adjuvant chemotherapy (rectal cancer radiotherapy, at least six cycles of CAPOX regimen, or at least eight cycles of FOLFOX6 regimen postoperative adjuvant chemotherapy). The DFS was evaluated as the primary end point. In addition, the patients' TCM symptoms and drug safety were evaluated as secondary indexes. The effect and safety of FZXJ were also evaluated.

### 2.5. Inclusion and Exclusion Criteria

The case inclusion criteria were as follows: (1) diagnosis of stage IIIC colorectal cancer according to the seventh edition American Joint Committee on Cancer (AJCC) staging criteria by histology or cytological pathology; after the initial screening, all of the enrolled patients were required to sign informed consent; (2) age ≥18 years, including both male and female patients; and (3) patients who underwent laparoscopic or open R0 resection and completed at least six cycles of CAPOX or eight cycles of FOLFOX6 postoperative adjuvant chemotherapy were assigned to their groups within 2 months of their last chemotherapy treatment, and no recurrence and metastasis were found in the random evaluation; (4) rectal cancer patients were included and allowed to receive perioperative radiotherapy (preoperative radiotherapy or chemotherapy to reduce lesion volume, or postoperative radiotherapy or chemotherapy alone to prolong the patient's life); (5) the subjects' general condition was good, meaning their Eastern Cooperative Oncology Group (ECOG) score was 0-2 and their expected survival time was more than 6 months; (6) patients having normal blood routine parameters and insignificant abnormalities in cardiac, liver, and kidney function were included.

Exclusion criteria were as follows: (1) pregnancy or lactation; (2) after the completion of adjuvant treatment, metastasis or recurrence occurred, as detected in imaging evaluation before the TCM treatment; (3) a history of symptomatic heart disease (arrhythmia, cardiac insufficiency, or myocardial infarction); (4) presence of an active infection, active bleeding, or severe metabolic disorder; (5) a history of other malignant tumors (unless they have been cured for more than 5 years); (6) patients undergoing other clinical drug trials or less than three treatment cycles after the end of the previous clinical drug trial; and (7) subjects judged by the researcher as not suitable for participation in the project.

Exit criteria/study termination criteria were as follows: (1) withdrawal of informed consent; (2) reaching the study end point (recurrence or death), intolerance, or loss to follow-up; (3) occurrence of serious adverse events (including grade 3 or 4 toxic and side effects defined in the CTCAE4.0 standard), where either the subject or the investigator considered it necessary to terminate the study; (4) disease recurrence or metastasis during treatment, according to the RECIST1.1 standard, confirmed by computed tomography (CT) or magnetic resonance imaging, or confirmed by cytology and pathology; (5) pregnancy occurred during treatment; (6) application of other antitumor chemicals or TCM during the treatment; and (7) poor compliance and unwillingness to continue participating in the clinical research, or selfinterruption of the treatment or follow-up.

### 2.6. Interventions

The interventions in this study for each group were as follows.

Treatment group: from the time of enrollment, the patients took the Chinese medicine (FZXJ) provided in this experiment for at least 6 months.

Basic prescription for FZXJ : Six Chinese medicines, namely, *Astragali Radix*, *Ganoderma*, *Atractylodis Macrocephalae Rhizoma*, *Coicis Semen*, *Herba Hedyotidis Diffuse*, and *Scorpion*. In addition, supplementary drugs were added according to the syndrome.

The use of drugs should be increased based on the following symptoms:

1. Asthenia (deficiency of vital energy): treating and tonifying the vital energy by adding *Polygonati rhizoma* and *Agrimoniae Herba*
2. Susceptibility to cold (*qi* deficiency and lack of firmness): tonifying the *qi* and strengthening the superficial by adding *Saposhnikoviae Radix*
3. Anorexia (weakness of the spleen and stomach): nourishing the spleen and stomach by adding *Gall Gigerii Endothelium*, *Crataegi Fructus*, and *Hordei Fructus Germinatus*
4. Epigastric distension (*qi* stagnation in the middle Jiao): treating *qi* stagnation by adding *Codonopsis Radix*, *Dioscoreae Rhizoma*, and *Euryales Semen*
5. Diarrhea (spleen dyskinesia): strengthening the spleen and helping in transportation by adding *Codonopsis Pilosula*, *yam*, and *Euryale Ferox*
6. Predawn diarrhea (deficiency of spleen and kidney *yang*): warming and tonifying the spleen and kidney by adding *Aconm Lateralis Radix Praeparaia*, *Myristicae Semen*, *Psoraleae Fructus*, and *Schisandrae Chinensis Fructus*
7. Defecation slippage not helpful (deficiency of spleen and kidney *yang*): treating to simulate warming *yang* and astringent intestines by adding *Halloysitum Rubrum*, *Granati Pericarpium*, *Galla chinensis*, and *Chebulae Fructus*
8. Constipation (fluid deficiency and intestinal dryness): moistening the intestines and defecation, senna, by adding *Cannabis Fructus* and *Pruni Semen*

Control group: the placebo was 1/10 of the prescription of FZXJ.

Both groups received granules twice a day, two packs each time.

### 2.7. Randomization

In this study, randomization was achieved by a computer-generated random number list prepared by an investigator with no clinical involvement in the trial.

### 2.8. End Point Assessments

The primary efficiency index included the patients' DFS. The disease assessment was based on the Response Evaluation Criteria In Solid Tumors (RECIST, V1.1). The TCM syndrome score was based on the “Chinese Medicine Treatment and Treatment Program for Colorectal Cancer” promulgated by the Chinese Medicine Administration. These include spontaneous symptoms such as fatigue, emotional depression, chest tightness, insomnia, anorexia, abdominal distension, abdominal pain, soreness, and weakness in the waist and legs, chills, and dysphoria in the chest, palm, and soles. Higher scores indicated more obvious symptoms (score range: 0, 1, 2, 3). Safety assessment included checking blood routine parameters, liver and kidney function indicators, and electrocardiogram results.

### 2.9. Traditional Chinese Medicine Curative Effect Evaluation Standard

For the effective rate, we mainly adopted the calculation method of score reduction rate and carried out symptom classification and curative effect evaluation with reference to the guiding principles for clinical research of new TCM. “Significantly effective” was defined when the score after treatment was reduced by ≥ 70% compared with that before treatment; “effective” was defined as the score after treatment being reduced by ≥ 30% and <70% compared with that before treatment; and “ineffective” was defined as being when there was no significant change in the score after treatment, or when the condition worsened.

### 2.10. Statistical Analysis

SPSS25.0 and R software were used for statistical analysis. The primary end point was DFS. The Kaplan–Meier curve was used for survival benefit assessment. *p* < 0.05 was considered statistically significant. The Chi-squared test was used to compare the curative effect between the two groups. No interim analysis was conducted in this trial. However, an independent statistician was allowed to access the database, continuously monitor the main adverse reactions, and report the results to the Safety Committee quarterly.

## 3. Results

### 3.1. Patients' Characteristics

We enrolled patients who received chemotherapy at the Department of Traditional Chinese Medicine, General Surgery, and Oncology of Shanghai Ruijin Hospital, from February 1, 2018 to February 28, 2022. These 150 patients were randomly assigned to the treatment group (*n* = 100, treated with FZXJ granule) and the control group (*n* = 50, treated with placebo). The demographic information of the patients (including gender and age), ECOG performance status, primary site, and postoperative adjuvant chemotherapy regimen were recorded in the complete analysis set. There was no significant difference in demographical information, primary site, and postoperative adjuvant chemotherapy regimen between these two groups of patients (*p* > 0.05). Therefore, these two groups were comparable (Table 1).

### 3.2. TCM Treatment Prolongs DFS

In this study, 12.6% of the patients eventually showed disease progression, including 9 cases in the control group and 10 cases in the treatment group. The DFS was 34.37 ± 2.91 months in the control group and 37.0 ± 1.08 months in the treatment group. There was a significant difference in the DFS between the two groups (*p* < 0.05) (Table 2, Figure 2).

### 3.3. Evaluation of the TCM Symptom Score in Both Groups

#### 3.3.1. Comparison of the TCM Symptom Score between the Two Groups

Before the treatment, the TCM syndrome scores of the two groups were similar. After treatment, compared with the control group, the treatment group showed less fatigue, abdominal distension, and soreness and weakness in the waist and legs (*p* < 0.05). The scores of emotional depression and anorexia decreased obviously, with a significant difference (*p* < 0.01). There were no significant differences in the incidence of chest tightness, insomnia, abdominal pain, chills, and dysphoria in the chest, palm, and soles between the two groups (*p* > 0.05) (Table 3, Figure 3).

#### 3.3.2. Effective Rate of TCM Symptoms

The statistics of the total effective rate in the control group revealed that there were 4 cases with significantly effective, 21 cases with effective, and 25 cases with ineffective treatment. In the treatment group, there were 24 cases with significantly effective, 47 cases with effective, and 29 cases with ineffective treatment. There was a significant difference between the two groups (*p* < 0.01) (Table 4, Figure 4).

### 3.4. Safety Evaluation

One patient in the control group developed lower extremity skin purpura after taking Chinese medicine granules for 1 month. However, we could not prove that the effect was related to FZXJ granules. None of the groups experienced any liver and kidney toxicity, indicating that Chinese medicine is safe and effective.

## 4. Discussion

In general, the 5-year total survival and DFS rate of patients with colorectal cancer after adjuvant chemotherapy are about 70%. The DFS rate of patients with stage III colorectal cancer is particularly low. Conventional chemotherapy is conducive to survival, but it has toxic side effects in the body. The incidence of severe adverse reactions such as vomiting, diarrhea, agranulocytosis, and peripheral neurotoxicity is as high as 5%-20% [13–16]. More importantly, after half a year of high-intensity chemotherapy, modern medicine enters an observation period with almost no treatment, which is the “window period” of treatment. Therefore, how to effectively and permanently inhibit tumor recurrence and ensure good tolerance of patients has been the focus of oncology research for a long period, which is also an urgent problem to be solved. It is also the focus of this research.

Professor Xiaoheng Shen defined the rehabilitation period after chemotherapy, where the body is in the recovery period and TCM treatment is dominant. Therefore, the pathogenesis of this period is that there is “the asthenia of the pathogens and the asthenia of the vital *qi*,” and Chinese medicine treatment is mainly used to support the healthy *qi*, supplemented by dispelling evil. The purpose is to support vital-*qi*, take care of middle energizer, and promote the body's recovery, supplemented by detoxifying and dispersing the knot to prevent cancer recurrence. The basic prescription for the rehabilitation period is composed of *Astragali Radix*, *Ganoderma*, *Atractylodis Macrocephalae Rhizoma*, *Coicis Semen*, *Herba Hedyotidis Diffuse*, and *Scorpion*.

FZXJ takes *Astragali Radix* and *Ganoderma* as monarch drugs; *Atractylodis Macrocephalae Rhizoma* and *Coicis Semen* are matched as ministerial medicines to tonify *qi*, invigorate the spleen, and eliminate dampness, so that the spleen and stomach can be recovered, and the middle jiao can be strengthened; *Herba Hedyotidis Diffuse* and *Scorpion* clear away heat and toxic materials, softening and dispersing hard masses into adjuvant drugs. Although *Herba Hedyotidis Diffuse* and *Scorpio* are cold, the combination of *Astragali Radix*, *Atractylodis Macrocephalae Rhizoma*, and *Coicis Semen* does no harm to the stomach caused by bitter cold. Although *Atractylodis Macrocephalae Rhizoma* is suspected of helping heat, it is restricted by *Herba Hedyotidis Diffuse* and *Scorpion*. All the herbs in Chinese medicine have the effects of invigorating *qi* and spleen, eliminating dampness, and resolving hard masses. The fundamental research showed that the activity of HT-29 cells and SW620 cell lines decreased after treatment with FZXJ granules, which could inhibit cell proliferation [17].

The results of this study showed that FZXJ granule effectively improved the main symptoms of patients, such as fatigue, abdominal distension, soreness and weakness in the waist and legs, emotional depression, anorexia, and prolonged DFS. Compared with the control group, the difference was statistically significant, indicating that FZXJ granule can effectively improve the symptoms and prolong the survival period of stage IIIC colorectal cancer patients.

In the future, we will incorporate more data to prove that the TCM treatment proposed in this project can prolong the DFS of patients with stage IIIC colorectal cancer and reduce the risk of recurrence and metastasis. After obtaining clear clinical evidence, we will establish and improve the “high-efficiency, low-toxicity, and individualized” integrated traditional Chinese and modern medicine diagnosis and treatment model for colorectal cancer [18] after adjuvant chemotherapy, form a diagnosis and treatment standard, and promote it.

## 5. Conclusion

In summary, FZXJ therapy can potentially be used to treat postoperative adjuvant chemotherapy patients with stage IIIC colorectal cancer. It can effectively improve patients' symptoms and prolong DFS. This maintenance treatment regimen is safe and effective and, therefore, can be applied in clinical practice.

## Figures and Tables

**Figure 1:** Experimental study flowchart.

**Figure 2:** Kaplan–Meier curve for DFS.

**Figure 3:** Comparison of TCM symptom score between the groups. The left graph shows the results before treatment, and the right graph shows the results after treatment.

**Figure 4:** Effective rate of TCM symptoms of the patients in both groups after treatment.

**Table 1:** Basic characteristics of patients.

Characteristic	Control group (*n* = 50)	Treatment group (*n* = 100)	*p* value
Sex	—	—	—
Male	37 (74%)	64 (64%)	0.218
Female	13 (26%)	36 (36%)	—

Age, years	—	—	—
Mean ± SD	63.14 ± 12.45	63.30 ± 12.90	0.942

Primary site	—	—	—
Colon	43 (86%)	78 (78%)	0.242
Rectum	7 (14%)	22 (22%)	—

Adjuvant chemotherapy	—	—	—
XELOX	43 (86%)	91 (91%)	0.350
FOLFOX	7 (14%)	9 (9%)	—

ECOG performance status	—	—	—
0	19 (38%)	29 (29%)	0.060
1	25 (50%)	67 (67%)	—
2	6 (12%)	4 (4%)	—

**Table 2:** Number of relapse and metastases and DFS in both groups.

Group	*N*	Relapse and metastases	DFS	*p* value
Control group	50	9 (18%)	34.37 ± 2.91	0.029
Treatment group	100	10 (10%)	37.0 ± 1.08	

**Table 3:** Comparison of TCM symptom score within and between the groups.

TCM symptom	Control group		Treatment group		*p* value
	Before treatment	After treatment	Before treatment	After treatment	After treatment
Fatigue	2.26 ± 0.69	1.36 ± 0.80	2.25 ± 0.80	0.99 ± 0.82	0.01
Emotional depression	1.9 ± 0.79	1.68 ± 0.77	1.97 ± 0.78	1.09 ± 0.96	0.005
Chest tightness	1.64 ± 0.85	1.18 ± 0.8	1.73 ± 0.84	1 ± 0.86	0.22
Insomnia	1.22 ± 0.82	1 ± 0.7	1.42 ± 0.96	0.92 ± 0.79	0.544
Anorexia	1.54 ± 0.93	1.12 ± 0.96	1.48 ± 0.96	0.65 ± 0.73	0.001
Abdominal distension	1.76 ± 0.85	0.96 ± 0.81	1.73 ± 0.81	0.63 ± 0.74	0.013
Abdominal pain	1.3 ± 1.02	1.02 ± 0.74	1.46 ± 0.98	1.12 ± 0.82	0.469
Soreness and weakness in the waist and legs	1.2 ± 1.05	1 ± 0.90	1.25 ± 1.04	0.67 ± 0.75	0.013
Chills	1.86 ± 0.78	0.98 ± 0.99	1.83 ± 0.91	1.03 ± 0.9	0.758
Dysphoria in the chest, palm, and soles	1.66 ± 0.85	1.08 ± 0.78	1.65 ± 0.87	1.01 ± 0.82	0.618

**Table 4:** Effective rate of TCM symptoms of the patients in both groups after treatment.

Group	*N*	Significantly effective	Effective	Ineffective	*p* value
Control group	50	4 (8%)	21 (42%)	25 (50%)	0.009
Treatment group	100	24 (24%)	47 (47%)	29 (29%)	

## Data Availability

The data used to support the findings of this study are included within the article.
